# Protective Effects of Pretreatment with Oleanolic Acid in Rats in the Acute Phase of Hepatic Ischemia-Reperfusion Injury: Role of the PI3K/Akt Pathway

**DOI:** 10.1155/2014/451826

**Published:** 2014-04-16

**Authors:** Bo Gui, Fuzhou Hua, Jie Chen, Zeping Xu, Hongbin Sun, Yanning Qian

**Affiliations:** ^1^Department of Anesthesiology, 1st Affiliated Hospital, Nanjing Medical University, Nanjing, China; ^2^Key laboratory of Anesthesiology, Xuzhou, Jiangsu, China; ^3^Department of Anesthesiology, 2rd Affiliated Hospital, Nanchang University, Nanchang, China; ^4^Department of Emergency, 1st Affiliated Hospital, Nanjing Medical University, Nanjing, China; ^5^Department of Anesthesiology, Jiangsu Tumor Hospital, Nanjing, China; ^6^Center for Drug Discovery, College of Pharmacy, China Pharmaceutical University, Nanjing, China

## Abstract

Oleanolic acid (OA) has been used to treat liver disorders, but whether it can attenuate hepatic ischemia-reperfusion- (IR-) associated liver dysfunction remains unexplored. In the present study, 160 male Sprague-Dawley rats were equally divided into five groups: group SH received neither hepatic IR nor drugs; group IR received hepatic IR without drugs; group CM and group OA received 0.5% sodium carboxymethylcellulose and 100 mg/kg OA, intragastrically, once a day for seven days before the hepatic IR, respectively; on the basis of treatment in group OA, group OA+wortmannin further received 15 *μ*g/kg of PI3K inhibitor wortmannin, intraperitoneally, 30 min before the hepatic IR. Then each group was equally divided into four subgroups according to four time points (preoperation, 0 h, 3 h, and 6 h after reperfusion). Serum ALT activity, IL-1*β* concentration, and hepatic phosphorylation of PI3K, Akt, and GSK-3*β* protein expression were serially studied. We found that OA pretreatment improved histological status and decreased serum ALT and IL-1*β* levels. It also increased p-PI3K, p-Akt, and p-GSK-3*β* protein expression at all the four time points. Prophylactic wortmannin partially reversed OA's protective effects. The data indicate that OA pretreatment protects liver from IR injury during the acute phase partially through PI3K/Akt-mediated inactivation of GSK-3*β*.

## 1. Introduction

Oleanolic acid (3*β*-hydroxy-olea-12-en-28-oic acid, OA) is a pentacyclic triterpene acid which exists naturally in vegetable oil, food, and some medicinal herbs [1]. OA provides protection against experimental hepatic injury in rats and has been used as an oral remedy for human liver dysfunction [2, 3]. Pretreatment with OA also considerably decreases augmentation of serum alanine transaminase (ALT) activity and hepatic centrilobular necrosis induced by chemical hepatotoxicants in mice [4, 5]. However, the molecular mechanisms of OA-mediated hepatic protection remain unclear.

Surgeries such as liver transplantation, partial hepatic resection, and hepatic tumor resection may result in hepatic ischemia-reperfusion (IR) injury, which correlates with clinical reduction of liver function [6, 7]. A pathological consequence of the cessation of hepatic blood supply, followed by reperfusion, is cellular damage within the ischemic areas, which induce formation of reactive oxygen species, release of proinflammatory cytokines, and hepatocyte necrosis, ending in liver dysfunction [8]. Despite the evidence of OA protection against myocardial or cerebral IR injury [9, 10], the potential for this compound to attenuate hepatic IR-induced injury remains unexplored.

Glycogen synthase kinase (GSK-3*β*) activity has recently been identified in a number of studies as crucial in the regulation of the inflammatory response [11, 12]. Its inactivation is also involved in indirubin-3′-oxime-induced protection against hepatic IR injury in rats [13]. Phosphatidylinositol-3-kinase (PI3K)/protein kinase B(Akt) dependent inhibition of GSK-3*β* activity plays an important role in the protective effects of carbon monoxide against hepatic IR injury [14]. These promising results prompted us to investigate the possible beneficial effects of OA pretreatment in rats submitted to partial hepatic IR. In a mechanistic approach, activation of the PI3K/Akt pathway in hepatic tissue was also evaluated.

## 2. Materials and Methods

### 2.1. Chemicals

OA (purity > 98%) was purchased from Guiyang Pharmaceutical Company. Sodium carboxymethylcellulose (CMC-Na) was purchased from SINOPHARM (Shanghai, China). Wortmannin was purchased from Sigma (St. Louis, USA) and dissolved in dimethyl sulfoxide. Antibodies were purchased from Cell Signaling (Boston, USA). All other chemicals were of highest purity commercially available.

### 2.2. Animal Care and Hepatic IR Procedure

After approval by the Institutional Animal Care and Use Committee at Nanjing Medical University (Nanjing, China), 160 male SPF Sprague-Dawley rats (230–250 g) were purchased from SLAC Laboratory Animal Co., Ltd. (Shanghai, China). They were maintained at a 12:12 h light: dark cycle and given water ad libitum.

Each rat was anesthetized with 2.5% isoflurane with a small rodent face mask. Partial hepatic ischemia was conducted by performing a midline laparotomy exposing the liver hilum, and subsequent clamping of portal structures to the left and median lobes with a microvascular clip, yielding 70% hepatic ischemia [15]. The abdomen was covered during the ischemic period. After 60 min of 70% hepatic ischemia, the clip was removed to initiate hepatic reperfusion. The abdominal cavity was stitched with 4-0 silk sutures. The rectal temperature was maintained at 37 ± 0.5°C with a warming pad throughout the surgical process. The rats were injected with buprenorphine (0.1 mg/kg s.c) for postoperative analgesia (five rats, three of them were from anesthetic accident and the remaining two rats from postoperative infection). Therefore, the survival rate in this study was nearly 97%.

The 160 rats were randomly but evenly assigned to one of five groups: rats that received a sham operation (SH group) were submitted neither to the clamping procedure nor to drugs; rats in the IR group underwent IR treatment without drug delivery; rats in the CM group received 0.5% CMC-Na once a day for seven days, followed by IR; and rats in the OA group received 100 mg/kg OA once a day for seven days [16], followed by IR; on the basis of treatment in group OA, group OA+wortmannin further received 15 *μ*g/kg of PI3K inhibitor wortmannin, intraperitoneally, 30 min prior to hepatic IR [17]. OA suspension (20 mg/mL) was made with 0.5% CMC-Na aqueous solution. With regard to daily substance delivery, SH and IR rats received 2 mL physiological saline, the CM group received 0.5% CMC-Na aqueous solution, and the OA group received OA suspension. Moreover, according to different time points for collecting serum and hepatic specimens, each group was further equally divided into the following four subgroups: preoperation (Prep), 0 h, 3 h, and 6 h after reperfusion.

### 2.3. Hepatic Histological Examination

Rat livers were collected 6 h after IR and were cut into small tissue blocks (about 1 cm in length, width, and height). After the blocks had been fixed with 10% buffered formalin solution, they were embedded in paraffin. Paraffin-embedded sections (10 *μ*m thick) were prepared as usual for histological examination after hematoxylin and eosin staining.

### 2.4. Measurements of Serum ALT Activity and IL-1*β* Concentration

Serum ALT activity and the concentrations of IL-1*β* were measured by using ALT assay kit (Jiancheng Bioengineering, Nanjing, China) and IL-1*β* ELISA kit (USCN, Wuhan, China), respectively. Blood was taken from the postcaval vein at the four aforementioned time points and then centrifuged for 10 min. ALT activity in the serum was determined as described previously and expressed as international units per liter (U/L) [18]. Production of IL-1*β* in the serum was measured by ELISA kit according to the manufacturer's instructions.

### 2.5. Western Blot Analysis

The rats were all sacrificed by decapitation at the four time points. The livers were quickly excised free from any adhering tissues. Total tissue extracts were obtained by lysing the liver in ice-cold RIPA buffer in the presence of a cocktail of protease inhibitors (Roche, Molecular Biochemicals, Mannheim, Germany) and phosphatase inhibitors (1 mM sodium fluoride and 1 mM sodium orthovanadate). After centrifugation, protein concentrations were quantified using the Bradford method, and 70 *μ*g of protein for each sample was subjected to 12% sodium dodecyl sulfate-polyacrylamide gel electrophoresis. After electrophoresis, the proteins were subsequently electrotransferred onto polyvinylidene difluoride membranes. The blots were blocked with 5% milk powder and 0.1% Tween 20 in 10 mM Tris-HCl (pH 7.5) at room temperature for 2 h and then incubated with rabbit anti-p-PI3K, p-Akt, Akt, p-GSK3*β*, and GSK3*β* (1 : 1000, 1 : 1000, 1 : 500, 1 : 1000, and 1 : 500, resp.) at 4°C overnight. After three washes with TBS-T, the blots were then incubated with horseradish peroxidase conjugated anti-rabbit secondary antibody at a dilution of 1 : 10,000 at room temperature for 1 h. The bound antibodies were visualized using an ECL system and exposed to X-ray films (Kodak, Rochester, NY, USA). The immunoblots were washed briefly and then incubated with a rabbit anti-GAPDH (1 : 2000) for 40 min at room temperature, followed by a horseradish peroxidase conjugated anti-rabbit antibody. GAPDH protein was then visualized and detected as the loading biomarker of proteins mentioned above.

### 2.6. Data Analysis

Statistical analysis was performed using GraphPad Prism (GraphPad Software, Inc., San Diego, USA; version 5.00). Data were expressed as means ± SD. For the analysis of normally distributed data, one-way analysis of variance was used followed by Dunnett's *t* multiple comparison tests. A *P* value < 0.05 was considered statistically significant.

## 3. Results

### 3.1. Inhibition of PI3K with Wortmannin Partially Reversed Protective Effects of OA on IR-Induced Hepatic Injury

Histologically, whereas necrotic areas were significantly decreased in the OA pretreated group at 6 h after reperfusion, the PI3K inhibitor wortmannin worsened the hepatic histological status (Figure 1). Biochemically, the IR procedure strikingly increased serum ALT activity at 3 h and 6 h after reperfusion, indicating that the partial hepatic IR model was established successfully (Figure 2; *P* < 0.05). At the same time points, pretreatment with 0.5% CMC-Na alone (group CM) did not affect serum ALT activity, indicating that CMC-Na, which was used as a suspending agent, had no effects on liver function. In contrast, rats pretreated with 100 mg/kg OA had drastically inhibited serum ALT activity at 3 h and 6 h after reperfusion (*P* < 0.05), which reflected protective effects of OA against IR-induced hepatic injury. When compared with group OA, inhibition of PI3K with 15 *μ*g/kg wortmannin increased serum ALT activity at 3 h and 6 h after reperfusion (*P* < 0.05). However, serum ALT activity at 3 h and 6 h after reperfusion in group OA+wortmannin was still lower than those in group IR and group CM (*P* < 0.05), suggesting that protective effects of OA involved only partially the PI3K pathway.

### 3.2. PI3K Inhibitor Wortmannin Partially Abrogated Protective Effects of OA on Serum IL-1*β* Concentrations

Serum IL-1*β* concentrations were increased following the IR procedure, not only at 0 h after reperfusion, but also at 3 h and 6 h after reperfusion in both IR and CM groups (Figure 3). However, these changes were markedly decreased by OA pretreatment (*P* < 0.05), indicating that OA exerted anti-inflammatory effects against systemic injury induced by partial hepatic IR. Furthermore, suppression of IL-1*β* concentrations by OA pretreatment actually emerged at 0 h after reperfusion, prior to the decrease in ALT activity. When compared with group OA, wortmannin increased serum IL-1*β* concentration at 0 h, 3 h, and 6 h after reperfusion (*P* < 0.05). However, the serum IL-1*β* concentration at 3 h and 6 h after reperfusion in group OA+wortmannin remained lower than those in group IR and group CM (*P* < 0.05).

### 3.3. OA Pretreatment Enhances PI3K, Akt, and GSK-3*β* Phosphorylation

To further evaluate the mechanism of OA-induced protective effects against IR-stimulated hepatic injury, we explored the levels of p-PI3K, p-Akt, total Akt, p-GSK-3*β*, and total GSK-3*β* protein expression (Figures 4, 5, and 6). There were no significant differences in the basal levels of total Akt and total GSK-3*β* protein expression among the four groups. The IR procedure was followed by increased p-PI3K, p-Akt, and p-GSK-3*β* protein synthesis at 3 h and 6 h after reperfusion (*P* < 0.05) whether rats were pretreated with CMC-Na or not. Furthermore, OA pretreatment significantly increased p-PI3K, p-Akt, and p-GSK-3*β* protein synthesis in IR-stimulated rat liver not only at preoperation, but also at 0 h, 3 h, and 6 h after reperfusion (*P* < 0.05). These results indicated that preoperative OA treatment was an important activator of the PI3K/Akt pathway.

## 4. Discussion

The present work demonstrated that pretreatment with 100 mg/kg OA could reduce the liver injury caused by partial hepatic IR, as indicated by histological improvement and significant decreases in both serum ALT activity and IL-1*β* level. These results were associated with a marked increase in p-PI3K, p-Akt, and p-GSK-3*β* protein expression, strongly suggesting that PI3K/Akt-mediated inactivation of GSK-3*β* may be involved in the protective effect of OA pretreatment towards IR-induced rat liver dysfunction. Inhibition of PI3K with 15 *μ*g/kg of wortmannin partially reversed the OA protective effects on IR-induced hepatic injury, which further supported the involvement of the PI3K/Akt pathway.

The rat model with 70% hepatic IR experienced severe hepatic injury without obvious mesenteric venous hypertension. Mesenteric congestion was avoided by allowing intestinal blood flow through right and caudate lobes, which led to a satisfactory survival rate despite substantial hepatic IR injury.

One major hallmark of hepatic IR is inflammation-induced hepatopathology [19, 20]. At ischemia stage, proinflammatory cytokines, such as IL-1*β*, were instantly released [21]. After reperfusion, neutrophils, triggered by proinflammatory cytokines, are further activated to cross the endothelial barrier and translocate into hepatic tissue [22]. Hepatic enzymes and reactive oxygen species are then released to aggravate the associated hepatic tissue injury [23–25]. OA exerts anti-inflammatory effects on lipopolysaccharide-induced inflammation by inhibiting hyperpermeability and leukocyte adhesion and migration [26]. It also exerts protective effects against hepatic injury by inducing antioxidant enzymes such as HO-1 [27]. Our results confirmed the development of liver injury by markedly elevated ALT activity and, indirectly, by IL-1*β* concentrations, whereas OA pretreatment considerably reduced the enhancement of ALT activity and IL-1*β* concentrations induced by IR. In addition, IL-1*β* concentrations were suppressed prior to the reduction of ALT activity, suggesting that systemic inflammatory responses induced by partial hepatic IR might be an important promoter for hepatic damage during the acute phase.

The PI3K/Akt pathway has an endogenous negative regulatory function, which limits proinflammatory mediators and chemotactic events by reducing neutrophil infiltration and production of cytokines [28–31]. However, the role of the PI3K/Akt pathway in the modulation of partial hepatic IR-induced injury was poorly understood. In our study, increased expression of the P13K/Akt pathway in the absence of OA may be a compensatory mechanism to counteract cytokine release following IR. The role of PI3K in a given signaling pathway is often examined by the use of pharmacological tools. The PI3K inhibitor wortmannin has been successfully used to clarify the physiological roles of PI3K pathway. In our study, wortmannin partially reversed the protective effects of OA as shown by worsening histological status and increasing serum ALT and IL-1*β* levels. Our results also showed that OA pretreatment was able to further markedly enhance phosphorylation of PI3K and Akt protein expression not only at the preoperative period, but also at 0 h, 3 h, and 6 h after reperfusion. This finding was consistent with previous studies which have reported that activation of the PI3K pathway protected organs against IR injury [32, 33].

When N-terminal Ser9 residue of GSK-3*β* is phosphorylated, the phosphate-binding pocket is occupied by an intramolecular interaction with the phosphorylated Ser9. This interaction considerably inhibits GSK-3*β* activity by changing the conformation of the catalytic site and also by preventing the binding of the primed substrate. The N-terminal Ser9 residue of GSK-3*β* is within the consensus sequence of the substrates for Akt. Thus, GSK-3*β* is one of the downstream targets of PI3K/Akt pathway [34]. Inactivation of GSK-3*β* may result in a decrease of proinflammatory cytokines [35]. A recent study has also shown that GSK-3*β* inactivation was involved in a propofol-induced protective effect against IR injury in an isolated guinea pig heart [36]. Our data showed that the changes in p-GSK-3*β* paralleled the alterations of serum ALT activity and IL-1*β* expression. These results also suggested that the PI3K/Akt-mediated inactivation of GSK-3*β* might play an important role in hepatoprotective action owing to OA pretreatment.

There are some limitations in our study. Firstly, we did not compare the OA effects on hepatic IR injury depending on whether the administration was done before or after IR. Indeed, although pretreatment with OA might exert protective effects in some selective hepatic surgeries, posttreatment may be more practical than pretreatment in clinical use since injury is unexpected. Secondly, PI3K inhibitor wortmannin only partially reversed the protective effects of OA on hepatic IR injury, so that further studies designed to investigate the overall mechanism of the OA protective effects are warranted.

## 5. Conclusion

Our data suggest that OA pretreatment exerts hepatoprotective effects in a rat model of hepatic IR, likely involving the PI3K, p-Akt, and p-GSK-3*β* pathways (see schematic flow of OA's role in decreasing hepatic IR injury in Figure 7). We think that these findings may pave the road for future innovative therapeutic strategies in the field of ischemia-reperfusion related liver injury.

## Figures and Tables

**Figure 1:** Effects of pretreatment with OA on partial hepatic IR injury evaluated by histological examination of rat liver tissue. The sections of the five groups were prepared at 6 h after reperfusion (HE, ×400). Arrows indicate necrotic areas of liver tissue.

**Figure 2:** Effects of pretreatment with OA on the activity of ALT in rats induced by partial hepatic IR. Data are represented as means ± SD (*n* = 8). *P < 0.05, compared with group SH. ^#^ *P* < 0.05, compared with group IR. ^Δ^ *P* < 0.05, compared with group CM. ^&^ *P* < 0.05, compared with group OA.

**Figure 3:** Effects of pretreatment with OA on the release of IL-1*β* in rats induced by partial hepatic IR. Data are represented as means ± SD (*n* = 8). *P < 0.05, compared with group SH. ^#^ *P* < 0.05, compared with group IR. ^Δ^ *P* < 0.05, compared with group CM. ^&^ *P* < 0.05, compared with group OA.

**Figure 4:** Effects of pretreatment with OA on p-PI3K (p85*α*) protein expression in rats induced by partial hepatic IR. Expression of p-PI3K (p85*α*) protein was detected by western blot analysis (a). The GAPDH protein expression was determined as the internal standard. These bands were quantified and analyzed (b). Data are represented as means ± SD (*n* = 8). *P < 0.05, compared with group SH. ^#^ *P* < 0.05, compared with group IR. ^Δ^ *P* < 0.05, compared with group CM.

**Figure 5:** Effects of pretreatment with OA on p-Akt (ser473) and Akt protein expression in rat induced by partial hepatic IR. Expression of p-Akt (ser473) and Akt protein was detected by western blot analysis (a). These bands were quantified and analyzed (b). Data are represented as means ± SD (*n* = 8). *P < 0.05, compared with group SH. ^#^ *P* < 0.05, compared with group IR. ^Δ^ *P* < 0.05, compared with group CM.

**Figure 6:** Effects of pretreatment with OA on p-GSK-3*β* (ser9) and GSK-3*β* protein expression in rats induced by partial hepatic ischemia-reperfusion (IR). Expression of p-GSK-3*β* (ser9) and GSK-3*β* protein was detected by western blot analysis (a). These bands were quantified and analyzed (b). Data are represented as mean ± SD (*n* = 8). *P < 0.05, compared with group SH. ^#^ *P* < 0.05, compared with group IR. ^Δ^ *P* < 0.05, compared with group CM.

**Figure 7:** Proposed schematic flow of OA's role in attenuating hepatic IR injury. IR procedure induces activation of PI3K cascades and then results in increases in IL-1*β* and ALT in the serum. OA can further activate these molecular changes at the PI3K/Akt signaling pathway and results in the decreased serum ALT activity and IL-1*β* concentration.
